The article "Development of Atorvastatin Calcium Biloaded Capsules for Oral Administration of Hypercholesterolemia" was retracted in 2023. Reasons: signs of a paper mill; suspected computer-generated content; unreliable results or conclusions; concerns about the data.

# Development of Atorvastatin Calcium Biloaded Capsules for Oral Administration of Hypercholesterolemia

**DOI:** 10.1155/2022/4995508

**Published:** 2022-05-16

**Authors:** Chitra Karthikeyini Senthilvel, Kavitha Karuppaiyan, Ananth Pothumani, Ananthi Vedharethinam, Ancy Wilfred Jose, Jamal Moideen Muthu Mohamed, Mohamed El Sherbiny, Hasnaa Ali Ebrahim, Mohamed El Shafey, Minilu Dejene

**Affiliations:** ^1^K. M. College of Pharmacy, Madurai 625107, Melur Road, Uthangudi, Tamil Nadu, India; ^2^Department of Pharmaceutical Technology, BIT Campus, Anna University, Tiruchirappalli 620024, Tamil Nadu, India; ^3^College of Pharmacy, Shri Indra Ganesan Institute of Medical Science, Tiruchirappalli 620012, Tamil Nadu, India; ^4^Department of Basic Medical Sciences, College of Medicine, AlMaarefa University, Riyadh 11597, P.O. Box 71666, Saudi Arabia; ^5^Department of Basic Medical Sciences, College of Medicine, Princess Nourah bint Abdulrahman University, Riyadh 11671, P.O. Box 84428, Saudi Arabia; ^6^Department of Anatomy and Embryology, Faculty of Medicine, Mansoura University, Mansoura 35516, Egypt; ^7^Physiological Sciences Department, Fakeeh College for Medical Sciences, Jeddah, Saudi Arabia; ^8^Department of Biotechnology, College of Biological and Chemical Engineering, Addis Ababa Science and Technology University, Addis Ababa, Ethiopia

## Abstract

The goal of this study was to develop atorvastatin (ATN) calcium biloaded, i.e., immediate release (IR) and sustained release (SR) capsules that would promote the quick onset of action and a better dissolution profile on both the IR and SR aspects. The IR granules were prepared by the wet granulation method, and an aqueous solubility study proved that the IR granules released the ATN within 25 min compared to the pure drug due to the addition of PEG and super disintegrants such as croscarmellose (CC) and crospovidone (CP). The sustained release nanoparticles (SR-NPs) were synthesized using a solvent evaporation technique and an optimal combination of hydrophilic and hydrophobic polymers. The addition of a hydrophobic polymer to a hydrophilic polymer delays drug release, resulting in a sustained and controlled release lasting up to 12 hours. The drug release of ATN from SR nanoparticles followed the Higuchi and Korsmeyer–Peppas models and had first-order kinetics (*r*2 = ???). Fourier transform infrared spectrophotometry, powder X-ray diffraction, and differential scanning calorimetric analysis were used to test the prepared biloaded capsules, and the results showed that there was no significant interaction between the polymers, excipients, and drug. The SEM and DLS analysis clearly demonstrated that drug particles in a continuous layer were enclosed by polymers at the nanoscale. To summarise, integrating both layers into a single capsule resulted in a superior release profile and patient compliance. Finally, prepared biloaded capsules were discovered to exhibit both an IR and an SR profile.

## 1. Introduction

Atorvastatin (ATN) is a synthetic lipid-lowering agent present as a calcium salt. ATN calcium belongs to the second generation of statins. ATN lowers plasma cholesterol and lipoprotein serum concentrations by inhibiting HMG-CoA reductase and, subsequently, cholesterol biosynthesis in the liver, and it increases the number of hepatic LDL receptors on the cell surface for enhanced uptake and catabolism of LDL. Production of LDL and the number of LDL particles are reduced by AC [1]. As per BCS classification, ATN calcium exhibits class II properties. The absolute bioavailability of AC is reported to be 12%, and only 30% of the drug is absorbed on oral administration [2]. Poor oral bioavailability of ATR (12%) is due to inadequate dissolution in the gastrointestinal tract, and it is mainly attributed to its low aqueous solubility (0.1 mg·mL^−1^) and its crystalline nature that leads to dissolution rate-limited. Enhancement of the dissolution rate for poorly soluble drugs in water to improve their oral bioavailability is a challenging task [3].

In current research, various strategies were adopted by the investigators to increase the solubility, dissolution, and bioavailability of ATN such as incorporation within inert water-soluble pharmaceutical excipients such as polyvinyl pyrrolidone and the addition of amphiphilic pharmaceutical excipients that contain both hydrophilic and lipophilic moieties in their structure. They are widely used in improving the physicochemical characteristics of drugs and increasing the solubility of sparingly soluble drugs [4]. A better drug release profile with immediate and sustained activity will definitely yield good bioavailability.

A single-layer tablet or capsule is not designed on both aspects of quick onset of action and sustained release. It can lead to errors in drug release and patient compliance issues. But in the bilayer concept, preplanned dose fixation is also possible in immediate release (IR) and sustained release (SR) which results in appropriate drug release profiles. So loading both layer IR and SR into a single capsule is an attractive and alternative to conventional dosage form. The loading dose in IR was prepared by the wet granulation method with the incorporation of PVP and superdisintegrants such as croscarmellose (CC) and crospovidone (CP). Maintenance dose as SR was formulated by combining both hydrophilic and hydrophobic polymers with a solvent evaporation method to promote better controlling drug release [5]. In both layers, an optimized concentration of PEG 6000 was added to increase wettability, solubility, and reduction in particle size (amorphous form) [6].

Both ethyl cellulose and HPMC polymer are widely used in sustained release formulations to control the dissolution rate of drugs. HPMC has fast gel forming characteristics and controls the initial release but also exerts a sustained release effect through strong viscous gel formation. Hence, the objective of the present investigation was to develop an oral formulation of biloaded capsules to achieve a quick onset of action and a prolonged therapeutic effect by sustaining the action [7]. This biloaded concept reduces the fluctuation in drug blood levels, frequency of dosing, and enhances convenience and compliance, resulting in a reduction in adverse side effects and overall health care costs.

## 2. Materials and Methods

### 2.1. Chemicals and Materials

Atorvastatin (ATN) calcium was obtained as a gift sample from Medopharm, Chennai, India. Hydroxypropyl methylcellulose (HPMC) and ethyl cellulose (EC) were obtained from Medopharm, Chennai (India), at free of cost. Polyethylene glycol (PEG 6000) was procured as a sample-gift from Matrix (India). Ethanol and methanol were procured through Merck in India, and other reagents (analytical grade) were purchased from SD Fine Chem (Bangalore).

### 2.2. Preparation of IR Granules

Weighed amounts of ATN drug, PEG, and disintegrants such as CC and CP were mixed geometrically with PVP paste which was added until the cohesive mass was obtained. The obtained mass was sieved through a 10# mesh and kept in a dryer at 60°C. Then, dried granules were reduced in size and sieved through 20# mesh [8]. From the resultant granules, talc and magnesium stearate were added.

### 2.3. Preparation of Sustained Release Nanoparticles (SR-NPs)

The SR-NPs nanoparticles were prepared by the solvent evaporation method followed by sonication. The weighed amount of ATN drug was dissolved in methanol and an appropriate quantity of HPMC K4 as per Table 1 and was dissolved in water. Then, the drug was slowly added to the aqueous phase of the polymer and continuous mixing was carried out until the drug was encapsulated. Then, the nanodispersion was probe sonicated for 60 sec with 70% amplitude by the probe sonicator and transferred to a rotary flask evaporator kept at 60°C and the speed was 80 rpm [9]. The resulting dried film yielded an ATN encapsulated NPs.

### 2.4. Solubility Studies

The saturation solubility measurements were assayed through ultraviolet absorbance determination at 245 nm using a Shimadzu UV-Visible spectrophotometer. Weighed amounts of AC (pure drug), IR granules, and nanoparticles equivalent to 20 mg of the drug were separately introduced into 25 mL conical flasks containing 10 ml of pH 6.8 phosphate buffer. The sealed flasks were agitated on a rotary shaker for 24 h at 37°C and equilibrated for 2 days. An aliquot was passed through a 0.1 *μ*m membrane filter (Millipore Corporation), and the filtrate was suitably diluted and analyzed on a UV spectrophotometer at 245 nm [10]. The mean results of triplicate measurements and the standard deviation were reported.

### 2.5. Drug Loading (DL) and Encapsulation Efficiency (%EE)

The resultant SR-NPs were then centrifuged at a rate of 10000 rpm for about 15 minutes towards separating the unentrapped drugs. Free drug in the supernatant liquid was determined by utilizing the UV-spectrophotometer at 245 nm. Methanol was utilized for the necessary dilution process, and the solution was then filtered [11]. The drug entrapment and loading was calculated from following formula:

(1) $$\begin{array}{c} EE\left(\%\right)=\frac{\left(\text{experimental ATN content}\right)}{\left(\text{theoretical ATN content}\right)\times 100}, \end{array}$$

(2) $$\begin{array}{c} DL\left(\%\right)=\frac{\left(\text{Weight of ATN}\right)}{\left(\text{Weight of SR}-\text{NPs}\right)\times 100}. \end{array}$$

### 2.6. In Vitro Drug Release

*In vitro* drug release studies were performed in an USP Type II dissolution apparatus (Electro Lab, India) with the paddle method at a rotation speed of 50 rpm. Dissolution was carried out both in acid media and neutral media using an equivalent of 20 mg of ATN. The volume and temperature of the dissolution medium were 900 ml at 37 ± 0.2°C, respectively. Samples were withdrawn at fixed times and were filtered and assayed through ultraviolet absorbance determination at 245 nm using a Shimadzu UV Visible spectrophotometer. In order to investigate the drug release mechanism from nanoparticle formulations, the percentage cumulative drug release data was fitted into mathematical models like first order, Higuchi's model, and the Korsmeyer–Peppas model. The mean results of triplicate measurements and the standard deviation were reported [11].

### 2.7. Solid State Characterization

#### 2.7.1. Fourier-Transform Infrared (FTIR) Spectroscopy

The FTIR study was used to evaluate drug and excipients interaction in IR as well as SR. KBr technique was used and pellets were prepared in the ratio of 1 : 50 [12]. Then, samples were examined using FTIR spectrophotometer in the wave number region of 4000–400 cm^−1^.

#### 2.7.2. Powder X-Ray Diffraction (PXRD) Analysis

The PXRD patterns of pure drug and immediate and sustained release formulations were obtained at room temperature using a Siemens Diffractometer D5000 (Siemens, Germany) with Ni-filtered Cu K*α* radiation. The 2*θ* scan range was 5–60° with a step size of 0.02°, and the scan speed was 3° per min [12].

#### 2.7.3. Differential Scanning Calorimetric (DSC) Analysis

The thermal properties of the powder samples were investigated with a PerkinElmer differential scanning calorimetry (DSC)-7 differential scanning calorimeter/TAC-7 thermal analysis controller with an intracooler-2 cooling system (PerkinElmer Instruments, USA). The amount of product to be analyzed shall range from 3 mg and be placed in perforated aluminium sealed 50 *μ*L pan [12]. Heat runs for each sample have been set from 40 to 200°C at 5°C·min^−1^, using nitrogen as the blanket gas (20 mL·min^−1^).

### 2.8. Computational Model for Compatibility

The components ethyl cellulose, hypromellose, polyethylene glycol, and ATN were downloaded from the publicly available PubChem domine as a .sdf format and the 3d structures were opened in the material studio and converted to .xsd format (Figure 1). To convert the molecule to stable form, the forcite module was used and the geometrical optimization process was performed using the COMPASS force field algorithm. The nonbonded (electrostatic and Vander Waals) energy was summation by the atom-based method. The blending character of the components ethyl cellulose, hypromellose, and polyethylene glycol with the drug ATN was analyzed through adsorption locator and blends binding energy protocol in BIOVIA Material Studio version 2017 [13]. The simulation module run learned that the formulation was mixed well and a stable solution with the ethyl cellulose, HPMC, PEG, and drug ATN. The hydrogen bond and *π-*alkyl interactions with the drug made the formulation compatible. Furthermore, geometrically optimized components EC, hypromellose, PEG, and ATN were filled inside the cubic (periodic boundary) box (like a beaker) to make an accurate model in the i*n silico* environment.

The blends mixing protocol was created to examine interaction pattern and mixing energies between the polymers and drug ATN. Blends calculation starts with a fine mixing task and the molecules, the optimized components loaded in the input window as a base and screen mixing role. The energy and bin width were set as 1000000 and 0.02 kcal·moL^−1^ with 10000 clusters of 20 iterations (Figure 1). The interacted 100 frames of the lowest energy complex were saved in the end. As a final run, the adsorption locator module was used to find the adsorbing sites of each interacted component. The same set of optimized components of the formulation were submitted as adsorbates, and the annealing task was set with 3 cycles and 15000/cycle.

### 2.9. Particle Size (PS) and Zeta Potential (ZP) Analysis

The PS analysis was performed using laser diffractometry (LD) using the Mastersizer (Malvern Instruments) for the volume distribution. Before measurement, the samples had to be diluted with deionized water to obtain a suitable concentration for measurement [14]. The ZP analysis was performed to estimate the stability of the nanosuspensions. The samples were diluted with deionized water with conductivity adjusted to 50 *μ*S/cm^2^ by the addition of sodium chloride before measurement (performed in triplicate).

### 2.10. Scanning Electron Microscope (SEM) Analysis

The diluted SR-NPs were examined under a scanning electron microscope (Zeiss, model EVO 18) to study the complete morphological classification [14]. The nanoparticles were then attached at the top of the SEM aluminium stubs with the carbon-tape and then they were coated with gold by utilizing a sputter oater (Electron Microscopy Sciences; 550X model). The SR-NPs were placed in the expansion chamber and the SEM images of different regions were obtained and investigated. The process was carried out at a high vacuum range of 300 mTorr and the whole SEM analysis was carried out at 10 kV (i.e., an accelerating voltage).

### 2.11. Characterization of Capsules

#### 2.11.1. Uniformity of Weight

The test was performed as stated in the Indian Pharmacopoeia and each capsule was weighed. Each capsule was then opened and, without losing any part of the shell, the contents were completely removed. Each capsule shell was then weighed. The weight of the contents is the difference between the two weights [15]. The procedure was followed for a total of 20 capsules, and the average weight was computed. The pharmacopoeia specifies that not more than two of the individual weights deviate from the average weight by 10%, and none deviates by more than 20%. The IR and SR layers were loaded into “3”-sized hard gelatin capsules (colour code: white-colored body and pink-colored cap).

#### 2.11.2. Disintegration Time (DT) and Drug Content (DC)

A basket and rack assembly were used to determine the disintegration time. The pharmacopoeia states that the disintegration time for hard gelatin capsules should not exceed 30 min [15]. Contents from six capsules were emptied into a mortar, the amount of capsule fill equivalent to a single dose (20 mg) was weighed, and the drug content of the capsules was determined in accordance with the procedure mentioned in IP.

#### 2.11.3. In Vitro Drug Release

One capsule was placed in a USP Type II dissolution apparatus (Electro Lab, India) with the basket method at a rotation speed of 50 rpm. Dissolution was carried out both in acid media and neutral media using an equivalent of 20 mg of ATN biloaded formulation and pure drug of AC. The volume and temperature of the dissolution medium were 900 ml at 37.0 ± 0.2°C, respectively. Samples were withdrawn at fixed times and were filtered and assayed [15].

## 3. Results and Discussion

### 3.1. Preparation of Biloaded Capsules

The IR granules were prepared by the wet granulation method. SR nanoparticles were prepared by solvent evaporation and the sonication method. Each capsule consists of 5 mg of AC as a loading dose (IR) and 15 mg of ATN as a maintenance dose (SR). The SR nanoparticles equivalent to 15 mg of drug and the IR granules equivalent to 5 mg of drug were mixed with lactose, talc, and magnesium stearate and were filled into 3 sizes of empty gelatin capsules to develop biloaded capsules (Figure 2). Preformulation studies such as angle of repose, Hausner ratio, and Carr's index were found to show that blending powder has good flow properties [16]. 75 mg of SR nanoparticles were utilized, equivalent to 15 mg of ATN, and 18 mg of IR granules, equivalent to 5 mg of ATN.

### 3.2. Docking Study

The table showed the geometrically optimized energy of the initial loaded molecules in the forcite protocol. The total energy (Table 2) of the components ethyl cellulose hypromellose, PEG, and ATN was optimized from 621543.264, 154789496.305, 8251.826, and 63463873110.065 to the level of 51.256, −34.461082, 10.321, and 64.638 Kcal/mol, respectively, to be naturally stable for further studies.

Energy-minimizing stable configurations of the components are placed in the cubic box to exemplify the interactions of each component. The blend algorithm disclosed that the mixing of the components in the abovementioned ratio was decent and well compatible (Table 3). The graph illustrated the energy (PEG) of components of the formulation at a level that was low and negative—1.5 kcal/mol specified that the formulated combination was stable due to multiple nonbonded interactions with each other (Figure 3). Emix and *χ* value of each component with drug is shown in table, which proved that ethyl cellulose, HPMC, and PEG negative value indicated the good mix with drug [17].

Finally, the adsorption locator module run algorithm exposed the interaction configuration of each component in the formulation. Ethyl cellulose formed one hydrogen bond and one conventional hydrogen bond with the -OH group of the ATN (Figure 4(a)), and the surface binding showed the complete adhering of the ethyl cellulose on the hydrophobic region of the ATN drug [18] (Figure 4(b)). The HPMC networked two bonds in both the end of ATN. The hydrogen atom of cycloring formed a bond with the etheric oxygen atom, and the aliphatic hydrogen of HPMC developed *π*-alkyl interaction with the phenylic ring of the ATN (Figure 4(c)).  Figure 4(d) showed that the negative region binding configuration with the ATN. Analysis of the PEG interaction with ATN showed one hydrogen bond with aminic hydrogen with oxygen atom of PEG in Figures 4(e)-4(f).

All three components formed multiple hydrogen bonds and *π-*alkyl interactions, which made the ATN mix with ethyl cellulose, HPMC, and PEG proper chemical configuration.

### 3.3. Solubility Studies

The solubility data relating to ATR, with different proportion of PEG are listed in Table 4. The drug-to-PEG ratio was optimized by measuring the percent solubility in mg·ml^−1^. A drug-to-PEG ratio of 1 : 2 had a significantly enhanced solubility enhancement compared with ATN.

Therefore, the optimal ratio of 1 : 2 was selected for the further preparation of IR and SR granules [19]. This optimized ratio gave an impact of solubility on IR and SR which is given in Table 5.

### 3.4. DL Efficiency

In this study, we found that the DL efficiency of nanoparticles was increased on drug concentration and polymer concentration increased [19]. It was also noticed that the combination of hydrophilic and hydrophobic polymers at a 1 : 1 ratio encapsulated the drug up to 87.5% which was more than that of using a single polymer. Optimized parameters such as selection of polymer, concentration of polymer, and solvent evaporation method yield better DL and good entrapment efficiency (Figure 5).

### 3.5. FTIR Outcome

The FTIR spectrum of the pure drug ATN and IR has shown similar peaks at 2887, 1653 cm^−1^, 1107.14 cm^−1^, 750.31 cm^−1^, and 844 cm^−1^. The SR nanoparticles spectrum showed the different peaks at 2970.38 cm^−1^, 1560.41 cm^−1^, 1369.46 cm^−1^, 947.05 cm^−1^, and 511.14 cm^−1^. It proved that the drug was encapsulated by polymers. IR and SR blending powder also not showed the any new peaks other than pure drug, IR and SR [20]. This FTIR study clearly proved that biloaded capsules containing material did not interact with each other, so there was no interaction between drug and polymers (Figure 6(a)).

### 3.6. PXRD Outcome

The XRPD data were collected for the pure drugs, immediate and sustained release formulations in order to investigate any changes in physical form after development process (Figure 6(b)). The X-ray diffractogram of ATR shows sharp and intense peaks at diffraction angles (2*θ*) of 16.88, 18.97, 19.12, 21.49, 23.20, and 26.25°, suggesting a typical crystalline pattern, but ATN in nanoparticles shows few peaks at 16.96, 18.36, 19.08, 23.22, and 42.43° with low intensity [10]. This proves that the crystallinity of ATR decreases as most of the drug gets converted to an amorphous form. IR granules exhibit multiple sharp but less intense Bragg peaks in their XRPD patterns related to their semicrystalline nature. The absence of sharp peaks in SR nanoparticles clearly proves that the drug was completely encapsulated by the polymer mixer of HPMC and EC.

### 3.7. DSC Outcome

This study provides the thermal characteristics and stability of drug and processed samples (IR and SR). The resultant data support the FTIR interpretation. In this analysis, an IR broad endothermic peak of 70–75°C and a sharp endothermic peak of 120°C in SR were obtained. All the peak values were similar to those of a pure drug [20]. So DSC thermogram of IR and SR showed there was no interaction between drug and excipients and drug and polymer (Figure 6(c)). It was not related with drug melting point. The shift DSC peaks showed the drug excipient interaction or changes in crystalline form.

### 3.8. ATN Release and Kinetics

The dissolution profile showed that SR nanoparticles were prepared by combined polymer releases of ATN 99.8% at the end of 12 h. Developed nanoparticles releases the drug for 12 hr in controlled manner (Figure 7(a)). In this study, individual polymer did not provide the sustaining effect for up to 12 hours. It may be due to the hydrophilic character of HPMC, and drug release retardation was controlled by gelling and swelling nature. But the combinations of polymers yield the good sustaining effect [21]. So this study clearly proved that 1 : 1 ratios of combined polymers (HPMC and EC) have the capacity to encapsulate the drug ATN completely and provide good release retardant properties. It was reported that in the bilayer concept, above 85% of the drug amount is released within 30 min from the IR layer.

In order to determine the mechanism of drug release of ATN from SR nanoparticle, the cumulative drug release was fitted for various kinetic models for first order, Higuchi, and Korsmeyer–Peppas plots, and the results were shown in Figures 7(b)–7(d). Both the SR nanoparticle loaded capsule formulations were found to have a high correlation to first order kinetics of 0.0.666 as well as obey Higuchi plot 0.913. The measured release rate constants as per the Korsmeyer–Peppas model were 0.678 and the coefficients “*n*” value of the Korsmeyer-Peppas equation was within the limit with a *r*^2^ value of 0.991, in which the drug release mechanism was found to be non-Fickian diffusion [22].

### 3.9. PS and ZP Measurements

The result of PS analysis yielding a nanoparticle population with a diameter 532 nm and a polydispersity index of 0.385 (Figure 8(a)). The ZP values give a measure of the long-term stability for the particulate systems. The investigated nanoparticles showed a value of about −9 mV which indicates good stability of the prepared formulation. For a physically stable suspension stabilized by electrostatic repulsion, a ZP of about ± 30 mV is required as a minimum. In a combined electrostatic and steric stabilization, a minimum of ± 20 mV will be sufficient [19]. The formulated nanoparticles showed a ZP value of −9 mv and a PS of 532 nm showed the NPs might be stable for long term (Figure 8(b)).

### 3.10. Morphology

The SEM study showed that prepared nanoparticles were at the nanolevel. It was proved by Figures 9(a) and 9(b) which showed the particle size at 300 nm. It was due to impact of solvent evaporation, probe sonication methods were adopted for preparing SR nanoparticles. It was also attributed to the addition of PEG which diminished particle size by reducing surface tension [20]. This PS reduction results in a significant increase in the solubility and dissolution rate and thus may improve the bioavailability of ATN. These observations were supported by DLS studies.

### 3.11. Evaluation of Capsules

The capsules showed an average weight of 95 ± 0.10 mg complied with the limits for consistency of weight as per Indian Pharmacopoeia. The capsules showed a DT of 3.5 min and thus complied with the limits for disintegration time as per Indian Pharmacopoeia. The ATN content of the capsules was found to be 99.15 ± 0.13%.

### 3.12. In Vitro Release of ATN

The *in vitro* release performance of the developed capsules of ATN was compared with pure ATN (20 mg) in both pH 1.2 buffer and pH 6.8 phosphate buffer. Dissolution data from the biloaded capsules (Figure 9(c)) show that 35% of the ATN calcium was released within the first 30 minutes. This drug release is attributed to the inclusion of the disintegrants CC, CP, and PEG which rapidly absorb water and swell leading to rapid disintegration of biloaded capsules and fast drug release. Then, encapsulated nanoparticles release the drug with a sustained effect until the period of 12 h. It releases the drug 99.2% at the end of 12 hours. This sustained release is due to the combination of hydrophilic polymer and hydrophobic polymer. It should be noted that the type of drug and concentration found in those studies are different, which might yield different results. Swelling of HPMC results in gel like formation and ethyl cellulose gives a release retardant effect [23]. During the process of dissolution, as soon as the drug and polymer particles come into contact with the dissolution fluid, a gel layer is formed. The gelatinous layer is the determining factor in the enhancement of the dissolution rate. From the Stokes–Einstein equation, the diffusion coefficient is inversely proportional to the viscosity of polymer forms around the drug particles. In biloaded capsules, the order of dissolution increased for IR rather than SR. SR nanoparticles retard the drug release up to 12 hours because of mixer of hydrophobic polymer (EC) into hydrophilic polymer (HPMC) used.

## 4. Conclusion

In this study, ATN biloaded capsules were successfully developed and evaluated. Release profiles have shown that biloaded capsules are able to deliver the drug via two different defined release mechanisms: immediate and sustained release. The dissolution profile proved that the biloaded concept is a good platform to promote the quick onset of action and prolonged action. Combining both IR and SR layers into a single capsule reduces the frequency of dose and improves patient compliance.

## Figures and Tables

**Figure 1:** Components of formulation packed inside the cubic box.

**Figure 2:** Formulation of biloaded capsules with IR granules and SR-NPs.

**Figure 3:** Blend mixing energy of the formulated components.

**Figure 4:** (a, b) Interactions of ethyl cellulose with ATN. (c, d) Interactions of HPMC with ATN. (e, f) Interactions of PEG with ATN. Left: hydrogen bond and right: surface binding of the complex.

**Figure 5:** DL efficiency of (a) single polymer and (b) combination of polymers.

**Figure 6:** (a) FTIR spectra, (b) PXRD pattern, and (c) DSC thermogram of IR, SR, IR-SR, and ATN.

**Figure 7:** (a) In vitro release profiles of ATN biloaded SR nanoparticles, (b) first order, (c) Higuchi's, and (d) Korsmeyer-Peppas release plot of SR-NPs preparation.

**Figure 8:** (a) PS distribution and (b) ZP measurement of SR-NPs.

**Figure 9:** SEM image of (a) surface particle with 500 nm, (b) surface particle with 500 nm, and (c) comparison of dissolution profile of ATN biloaded capsules with pure ATN.

**Table 1:** Composition of IR granules and SR-NPs.

Layers	Ingredients (mg)						
	ATN	PEG	CC	CP	PVP	HPMC	EC
IR	5	10	1	1	1	—	—
SR-NPs	15	30	—	—	—	15	15

ATN, atorvastatin; CC, croscarmellose; CP, crospovidone; PVP, polyvinyl pyrrolidone; HPMC, hydroxy propyl methyl cellulose; EC, ethyl cellulose.

**Table 2:** Minimized energy of the components.

Energy contributor	Ethyl cellulose	Hypromellose	PEG	ATN
Total energy	51.256	−34.461082	10.321	64.638
Valence energy	−7.845	−39.120	0.212	180.903
Bond	3.495	7.319	0.013	9.030
Angle	26.171	37.840	0.042	28.565
Torsion	−37.510	−84.279	0.157	141.902
Inversion	0.0	0.0	0.0	1.406
Valence energy	−14.435	−19.909	0.0	−14.280
Stretch-stretch	0.087	0.209	0.0	0.159
Stretch-bend-stretch	−1.134	−1.634	0.0	−2.829
Stretch-torsion-stretch	−0.098	−0.063	0.0	−3.541
Separated-stretch-stretch	0.0	0.0	0.0	0.178
Torsion-stretch	−0.703	−0.465	0.0	−11.348
Bend-bend	0.192	0.069	0.0	0.171
Torsion-bend-bend	−5.743	−7.456	0.0	−0.763
Bend-torsion-bend	73.535	−10.568	0.0	3.692
Nonbond energy				−101.985
Van der Waals	5.507	0.196	−0.076	16.049
Electrostatic	68.029	24.371	10.186	−118.034

**Table 3:** Mixing energy value and *χ* value of each components.

Base	Screen	Chi (298 K)	Emix (298 K)
ATN	Ethyl cellulose	−99.7926	−59.096
ATN	Hypromellose	−145.746	−86.309
ATN	PEG	−137.591	−81.4798

**Table 4:** Ratio optimization of ATN to PEG.

Drug: PEG	% Solubility enhancement
1 : 0.5	40.18^*∗*^
1 : 1	55.3^*∗*^
1 : 1.5	70.35^*∗∗*^
1 : 2	80.32^*∗∗*^

**Table 5:** Solubility studies of ATN (mean ± standard deviation) from IR and SR in comparison with pure ATN.

Product	Solubility (mg·mL^−1^)
ATN calcium	0.15
SR-NPs	0.5^*∗∗∗*^
IR	0.82^*∗∗∗∗*^

*n* = 3; *P* < 0.05; ^*∗∗∗∗*^refers to significant difference amongst treatment groups.

## Data Availability

The datasets used and/or analyzed during the current study are available from the corresponding author on reasonable request.
